# Utilization of Ultrasonic Image Characteristics Combined with Endoscopic Detection on the Basis of Artificial Intelligence Algorithm in Diagnosis of Early Upper Gastrointestinal Cancer

**DOI:** 10.1155/2021/2773022

**Published:** 2021-11-29

**Authors:** Liang Wang, Hui Song, Ming Wang, Hui Wang, Ran Ge, Yan Shen, Yongli Yu

**Affiliations:** ^1^Digestive Endoscope Room, Cangzhou Central Hospital, Cangzhou 061001, Hebei, China; ^2^Department of Gastroenterology, Cangzhou Central Hospital, Cangzhou 061001, Hebei, China; ^3^Department of Tumor Radiotherapy, Cangzhou Central Hospital, Cangzhou 061001, Hebei, China

## Abstract

The aim of this study was to evaluate the diagnostic value of artificial intelligence algorithm combined with ultrasound endoscopy in early esophageal cancer and precancerous lesions by comparing the examination of conventional endoscopy and artificial intelligence algorithm combined with ultrasound endoscopy, and by comparing the real-time diagnosis of endoscopy and the ultrasonic image characteristics of artificial intelligence algorithm combined with endoscopic detection and pathological results. 120 cases were selected. According to the inclusion and exclusion criteria, 80 patients who met the criteria were selected and randomly divided into two groups: endoscopic examination combined with ultrasound imaging based on intelligent algorithm processing (cascade region-convolutional neural network (Cascade RCNN) model algorithm group) and simple use of endoscopy group (control group). This study shows that the ultrasonic image of artificial intelligence algorithm is effective, and the detection performance is better than that of endoscopic detection. The results are close to the gold standard of doctor recognition, and the detection time is greatly shortened, and the recognition time is shortened by 71 frames per second. Compared with the traditional convolutional neural network (CNN) algorithm, the accuracy and recall of image analysis and segmentation using feature pyramid network are increased. The detection rates of CNN model, Cascade RCNN model, and endoscopic detection alone in early esophageal cancer and precancerous lesions are 56.3% (45/80), 88.8% (71/80), and 44.1% (35/80), respectively. The detection rate of Cascade RCNN model and CNN model was higher than that of endoscopy alone, and the difference was statistically significant (*P* < 0.05). The sensitivity, specificity, positive predictive value, and negative predictive value of Cascade RCNN model were higher than those of CNN model, which was close to the gold standard for physician identification. This provided a reference basis for endoscopic ultrasound identification of early upper gastrointestinal cancer or other gastrointestinal cancers.

## 1. Introduction

Early gastrointestinal cancer refers to early gastrointestinal tumor [1]. Most patients have no special symptoms and are often found in high-risk people over the age of 40. High-risk people refer to long-term gastrointestinal diseases or gastrointestinal tumors in immediate relatives [2]. The digestive tract includes the mouth, throat, esophagus, stomach, duodenum, small intestine, colon, and rectum. Esophageal cancer (EC) is a clinical malignant tumor, which is mostly seen in men over 40 years old [3]. Because there are no typical symptoms in the early stage of esophageal cancer, the sensitivity of patients to esophageal cancer is not high. Most patients with esophageal cancer are already in the advanced stage of gastrointestinal cancer. The mortality rate of advanced cancer is very high, and a large number of anticancer measures make patients miserable. The survival rate of patients with early gastrointestinal cancer after surgical resection is high, but the survival rate of elderly patients is low because of weak physique and other elderly diseases [4]. Early esophageal cancer only affects the submucosa and can be treated by minimally invasive surgery under ultrasonic endoscopy. Its surgical effect is good, which can almost achieve the effect of surgery and improve the detection rate and diagnosis rate of early esophageal cancer [5]. If esophageal cancer can be treated at an early stage, it will be of great benefit to the future treatment and prognosis of patients and can also reduce the cost burden of patients, which has great clinical significance for the treatment of cancer [6].

The digestive tract is divided into upper digestive tract and lower digestive tract. The upper digestive tract refers to the digestive tract including esophagus, stomach, and duodenum [7]. The lower digestive tract generally refers to the ileum. It is very common to use endoscopy to deal with digestive tract diseases. The upper digestive tract endoscopy usually refers to gastroscope, and the lower digestive tract endoscopy mainly refers to colonoscopy [8]. Deep learning technology has made a breakthrough in recent years. It has gradually become a hot research direction in the field of image processing and machine learning. Deep learning algorithm refers to a series of algorithms developed from artificial neural network. Compared with the traditional artificial neural network, the deep learning algorithm greatly strengthens the width and depth of the network. A large number of layers in the network can be responsible for feature extraction at different depths. From the extraction of line and edge information in the shallow layer of the image, to the extraction of the approximate shape of the target in the middle layer, and then to the extraction of deeper semantic information, deep learning can be competent. With these advantages, deep learning technology has been widely used in the field of image processing. As an important means of clinical diagnosis and treatment of digestive tract diseases, digestive tract endoscopy mainly uses camera and video to capture the internal state of digestive tract [9, 10]. However, the captured video and image quality may cause serious artifacts and blur, such as patient movement [11]. The amount of light can cause exposure or too much darkness, which will affect the image quality, resulting in specular reflection or pixel oversaturation [12]. Generally, endoscopic image interference occurs in different frequencies and modes. These interferences not only affect the observation of doctors for diagnosis and treatment but also cause misjudgment for artificial intelligence recognition [13, 14]. In addition, if the image interference can be detected correctly, it is of great significance to develop algorithms and interference repair algorithms.

In this study, the ultrasonic image characteristics combined with endoscopic detection in the diagnosis of early upper gastrointestinal cancer are studied. The research is suitable for the application of digestive endoscopy in the diagnosis of early upper gastrointestinal cancer. In this study, cascade region-convolutional neural network (Cascade RCNN) model is used for medical images of early gastrointestinal cancer. The images are identified and processed to find the lesions earlier, which provides a basis for the early treatment of early gastrointestinal cancer. The innovations of this part are as follows: considering the adjacent distribution and overlap of endoscopic image interference, the Cascaded CNN structure is combined with the feature pyramid network for extracting multiscale features to obtain larger features and improve detection performance, and a soft nonmaximum suppression algorithm is introduced.

## 2. Methods

### 2.1. Research Object

The source of cases was 120 inpatients in the hospital from June 2017 to June 2021. According to the inclusion and exclusion criteria, 80 patients who met the criteria were selected. Endoscopy was combined with ultrasonic imaging based on intelligent algorithm processing (Cascade RCNN model algorithm group) and endoscopy alone group (control group).

Inclusion criteria were as follows: (1) patients with esophageal lesions suspected by endoscopy, such as rough esophageal mucosa, patchy congestion, erosion, ulcer, small bulge, mucosal injury, abnormal color, or vascular texture changes; (2) patients over 18 years of age who can normally communicate and describe symptoms; (3) patients who had a history of early upper gastrointestinal cancer, are not cured, and are still observed and treated in the inpatient department.

Exclusion criteria were as follows: (1) patients with thyroid function injury; (2) patients with other upper gastrointestinal diseases; (3) patients with pregnancy, lactation, or planned pregnancy; (4) patients allergic to cephalosporin or other antibiotics; (5) patients with severe liver dysfunction; (6) patients under 25 years old.

In this study, 80 patients with early upper gastrointestinal cancer met the above inclusion criteria and exclusion criteria. This study was approved by the medical ethics committee of the hospital, and the family members of the patients included in the study signed the informed consent form.

### 2.2. Cascade RCNN Model

Convolutional neural networks (CNN) are a kind of feedforward neural networks with depth structure including convolution calculation. It is one of the representative algorithms of deep learning. CNN has the ability of representation learning and can carry out shift-invariant classification of input information according to its hierarchical structure. Therefore, it is also called “shift-invariant artificial neural networks (SIANN).” The Cascade RCNN model used in this study has evolved from CNN model. It consists of three main parts: feature extraction module, candidate region generation module, and detection module [15].  Figure 1 shows the network framework of Cascade RCNN. The feature extraction module consists of two parts. In addition to ResNet50, which is generally used as a basic network in the field of image classification, the feature pyramid network is also used to extract multiscale and multidimensional images. Therefore, the network can completely use low-level detailed features and high-level meaning information to improve the performance of target lesion detection rate (especially small lesion detection). The candidate region generation module is implemented by the candidate region generation network. After pyramid analysis, 15 locking frames with different sizes and aspect ratios will be generated. After locking the number of frames and pixel calculation, the effective candidate region is obtained by the soft nonmaximum suppression algorithm for the next classification and regression. The detection module uses the IoU threshold different from the three-level cascade structure to realize the classification of the generated candidate region and the accurate positioning of the boundary box. With this structure, when the cross ratio increases, the steep reduction of image accuracy can be effectively prevented.

As shown in Figure 2, feature pyramid networks (FPN) were applied to extract multidimensional and multiscale images. By changing the connection mode, the performance of medical image detection can be greatly improved without increasing the amount of calculation of the original model. FPN was a product of traditional CNN enhancement, which represented output image information. The feature extraction method of CNN was improved, and the final output feature can better represent the input image information of all dimensions. Based on the traditional CNN model, FPN developed an effective multidimensional feature representation method of input image by using the representation structures of different dimensions of images with the same scale. This can provide the basis for target detection and other tasks in the next stage, so as to produce more result graphs. Figure 2 shows the network structure.

As shown in Figure 3, FPN modified the original high-threshold risk, which would lead to the deviation of the final result. The cascaded regional CNN was used to connect each regression network to improve the image threshold. Cascade structure consisted of three serial detectors. Each detector was based on different IoU thresholds. The output of the former detector was used as the input of the latter detector, and the latter the detector, the greater the threshold. In this way, the detector at each stage can focus on detecting the candidate boxes of IoU in a certain range, and the detection effect will be better and better.

### 2.3. Endoscopic Examination Method

All cases were examined by a doctor with rich experience in endoscopic operation and senior professional title. Before the examination, the patient fasted and underwent water deprivation for 8–10 hours to confirm whether there were contraindications. 20–30 minutes before the examination, the patient took dyclonine hydrochloride mucilage orally and was left in lying position, with both lower limbs in flexion position and the mandible slightly raised to make the patient's esophagus entrance and oropharynx in the same straight line, so as to facilitate the insertion of endoscope, establish venous access, and give propofol (1.0-2.0 mg/kg) for intravenous anesthesia. After the endoscope enters the digestive tract and retreats to the esophagus, abnormal lesions were found, the location, size, and shape of lesions were recorded, and the esophageal mucosa and blood vessels were observed while retreating. The suspicious lesions of esophagus were observed carefully, and the location, size, and shape of the lesions were recorded.

### 2.4. Ultrasonic Examination Method

Ultrasonic examination method: the patient was routinely anesthetized on the oropharyngeal surface and injected with sterile water through the biopsy hole, and a 20 MHz ultrasonic probe was inserted. The scan was started after the cavity of the lesion was filled with water, and the lesion and its surrounding area at multiple levels were continuously scanned. Two senior and experienced endoscopists jointly judged the infiltration level of the lesion.

### 2.5. Pathological Acquisition

Pathology was obtained and sent for examination through endoscopic mucosal resection, mucosal dissection, or surgical treatment. The specific basis for selecting the treatment plan was mainly the ultrasonic characteristics of the medical focus in the ultrasonic endoscope, the source level, location, size, and so on. The specimens obtained through these schemes were further fixed by methylase, alcohol gradient dehydration, paraffin embedding, routine section, and staining, and the diagnosis was obtained combined with pathology.

### 2.6. Performance Evaluation of Detection Model

Precision (Pre), Dice similarity coefficients (DSC), and recall (Rec) are used to evaluate the algorithm effect of the model. The equations are as follows:

(1) $$\begin{array}{c} \mathrm{Pre}=\frac{\mathrm{TP}}{\mathrm{TP+FP}},\\ \mathrm{Rec}=\frac{\mathrm{TP}}{\mathrm{TP+FN}},\\ \mathrm{DSC}=\frac{\mathrm{2TP}}{2^{*}\mathrm{TP+FN+FP}}=\frac{\mathrm{2*Pre*Rec}}{\mathrm{Pre+Rec}}. \end{array}$$

TP represents the number of true positive pixels, FP represents the number of false positive pixels, and FN represents the number of false negative pixels. DSC can compare the excellent performance of the two algorithms and can also evaluate whether an algorithm meets the expected effect, with the doctor's judgment as the gold standard.

### 2.7. Experimental Platform

The hardware platform used for testing in this study is a deep learning server with RAM of 128G, and its display card is RTX2080Ti. The deep learning platform is based on TensorFlow keras, TensorFlow version is 1.14.0, and keras version is 2.2.4.

### 2.8. Statistical Methods

SPSS20.0 was used for analysis and statistics. The measurement data of normal distribution were expressed as mean ± standard deviation. One-way analysis of variance was used for intergroup comparison. The general data were compared by independent sample *t*-test and comparison of aneurysm occlusion at different time points in control group was performed by paired sample *t*-test. *P* < 0.05, and the difference was statistically significant.

## 3. Results

### 3.1. Visual Evaluation Segmentation Effect

The endoscopy and ultrasound images were obtained. CNN model and Cascade RCNN model were used to identify the lesions of early cancer of upper gastrointestinal tract. Comparing the ultrasound image based on neural network recognition algorithm with the doctor's manual recognition image, the doctor's manual recognition was clear and accurate. The RCNN image was close to the gold standard for doctor's recognition, but the reflective and shaded parts were identified as lesions in the endoscopic image. Compared with CNN model, RCNN model recognition had high recognition accuracy. CNN recognized a large number of highlights and shadows as early cancer features. RCNN had fewer recognition errors and was close to the gold standard for doctor recognition, as shown in Figures 4 and 5.

### 3.2. Comparison of the Efficiency of Two Algorithms in Identifying Early Gastrointestinal Cancer

The purpose is to use intelligent algorithms to distinguish and segment early esophageal cancer and normal tissues. The evaluation indicators use three indicators, precision, recall, and DSC, to comprehensively evaluate the performance of the model. The larger the value of these indicators, the better the segmentation performance of the network. During training, except for different model structure, activation function, and loss function, other superparameter settings are the same, the learning rate is 0.001, the batch size is 4, and the number of training times is 15,000, as shown in Figures 6–8.

Compared with the traditional CNN algorithm, the accuracy and recall and DSC of image analysis and segmentation using RCNN are increased. The accuracy of CNN was 0.7413 and that of Cascade RCNN model was 0.7982 (*P* < 0.05). The recall rate of CNN was 0.662 and that of Cascade RCNN model was 0.763 (*P* < 0.05). Moreover, the operation speed of Cascade RCNN model was significantly improved, which was closer to the requirements of real time in practical application. The prediction speed of CNN was 113 frames/s and that of Cascade RCNN model was 42 frames/s (*P* < 0.05). The results of learning efficiency, iteration, and prediction speed were shown in Figures 9–11.

### 3.3. Detection of Early Upper Digestive Tract Carcinoma and Precancerous Lesions in Two Groups

Figure 12 is the ultrasonic image feature map and endoscopic examination map of patients with early gastrointestinal cancer after artificial intelligence segmentation. The detection efficiency of the two groups is shown in Figures 13–19. 55 lesions were detected under CNN model, 75 lesions were detected under Cascade RCNN model, and 78 lesions were detected by endoscopy alone. The detection rates of CNN model, Cascade RCNN model, and endoscopy alone in early esophageal cancer and precancerous lesions were 56.3% (45/80), 88.8% (71/80), and 44.1% (35/80), respectively. The detection rate of Cascade RCNN model and CNN model was higher than that of endoscopy alone, and the difference was statistically significant (*P* < 0.05). The detection of early esophageal cancer and precancerous lesions by Cascade RCNN model was similar to that of endoscopy alone, and there was no significant difference between them (*P* > 0.05).

The sensitivity, specificity, positive predictive value, and negative predictive value of early esophageal cancer and precancerous lesions in the observation group and CNN group were significantly higher than those in the control group (*P* < 0.05). The sensitivity, specificity, positive predictive value, and negative predictive value of early esophageal cancer and precancerous lesions in the observation group and CNN group were similar (*P* > 0.05).

## 4. Discussion

Early upper gastrointestinal cancer is still a difficult cancer problem to overcome all over the world. The initial symptoms of early upper gastrointestinal cancer are not obvious, but cancers with other causes or other wrong findings in gastrointestinal endoscopy may have existed for a long time [16]. However, most of the early upper gastrointestinal cancers have symptoms such as difficulty to diagnose tumor progression. According to the data, only 1 of the 8 early upper gastrointestinal cancers was detected early [17]. After surgical resection of early esophageal squamous cell carcinoma, the 5-year survival rate of patients is as high as 85%–90%. Early detection, early diagnosis, and early treatment are very important to improve the prognosis of patients. Although the initial prognosis is good, it is difficult to find cancer-related indicators or lesions with color changes. In the previous ultrasonic endoscope images, it is not easy to observe the changes of upper gastrointestinal vessels, which easily causes misdiagnosis. In addition, endoscopy often generates multiple images. There are many applications of deep learning in medical image recognition. For example, Yang and Bang [18] used *k*-nearest neighbor classification algorithm to classify the features of enlarged endoscopic images, so as to recognize polyp images. El Hajjar and Rey [19] used support vector machine (SVM) classification algorithm to classify the features of enteroscopy images to realize the recognition of polyp images. Deep learning algorithms can often be regarded as a complete “end-to-end” system, so this kind of recognition method directly uses the convolution layer at the front end of the deep network to extract features and uses the output layer at the back end to classify them, so as to realize the recognition of lesion images. For example, Parasher et al. [20] used GoogLeNet to extract features and classify gastrointestinal images at the same time. Veitch et al. [21] used classical CNN to realize feature extraction and classification of narrow-band imaging enteroscopy images to identify colon polyp images.

In this study, a method combining Cascade RCNN and Cascade RCNN network is proposed. The principle of cascaded object detection framework is introduced, and the effectiveness of Cascade RCNN for multiscale feature extraction is discussed. When detecting endoscopic image detection, nonmaximum suppression algorithm is used to adjust the data filtering strategy to obtain better detection effect. The results of this study show that, compared with the ultrasonic image based on neural network recognition algorithm, the doctor's manual recognition image is clear and accurate. RCNN image is close to the gold standard of doctor recognition, and the RCNN recognition error is less, which is close to the gold standard of doctor recognition. Compared with the traditional CNN algorithm, the accuracy, recall, and DSC of RCNN segmentation are increased. The accuracy of CNN is 0.7692, and that of Cascade RCNN model is 0.7982, with an increase of 0.029 (*P* < 0.05). Recall of CNN is 0.662, and that of Cascade RCNN model is 0.763, with an increase of 0.101 (*P* < 0.05). DSC of CNN is 0.701, and that of Cascade RCNN model is 0.846, with an increase of 0.145 (*P* < 0.05). Cascade RCNN model more predicts the background (i.e., nonlesion area) as lesion area, the false detection rate increases slightly, and the larger monitoring area means that the missed detection rate decreases. The loss function is used to solve the problem of uneven classification distribution of conflict database. Experimental results showed that the proposed method was effective, the detection performance was better than CNN model algorithm, the results were close to the gold standard of physician recognition, and the detection time was greatly shortened.

This study proposes an image detection algorithm of early gastrointestinal cancer based on deep learning, which can accurately detect the lesions of early gastrointestinal cancer and suggest that the corresponding areas belong to the characteristics of early cancer to a certain extent. It is helpful for the followup development of computer-aided diagnosis method of gastrointestinal diseases, endoscopic image quality evaluation algorithm, and the diagnosis of other gastrointestinal diseases. Limitations of this study: the target detection network model used is still large and the detection speed is relatively slow. The model needs to be further optimized. In addition, the detection accuracy also needs to be further improved in order to better meet the needs of practical application. The data set used in this study is not large enough, and more samples need to be used to be tested in the future. Future research can develop more practical detection algorithms according to the detected medical images, which will be more helpful to the detection of gastrointestinal diseases.

## 5. Conclusion

This study shows that the ultrasonic image combined with endoscopic detection of artificial intelligence algorithm is effective, the detection performance is better than the traditional CNN model algorithm and endoscopic detection alone, and the detection time is greatly shortened. Compared with the traditional CNN algorithm, the accuracy, recall, and DSC of image analysis and segmentation using Cascade RCNN model are increased. The detection rates of CNN model, Cascade RCNN model, and endoscope alone in early esophageal cancer and precancerous lesions are 56.3% (45/80), 88.8% (71/80), and 44.1% (35/80), respectively. The detection rate of Cascade RCNN model and CNN model were higher than that of endoscopy alone, and the difference was statistically significant (*P* < 0.05). The sensitivity, specificity, positive predictive value, and negative predictive value of Cascade RCNN model were higher than those of CNN model and endoscopy alone, which was close to the gold standard for physician identification and provided a reference basis for ultrasonic endoscopy identification of early upper gastrointestinal cancer or other gastrointestinal cancers.

## Figures and Tables

**Figure 1:** Structure of Cascade RCNN model.

**Figure 2:** FPN network structure.

**Figure 3:** Cascade structure diagram.

**Figure 4:** Upper gastrointestinal endoscopy. (a) Doctor manually identifies early cancer lesions. (b) CNN model identifies early cancer lesions. (c) Cascade RCNN identifies early cancer lesions.

**Figure 5:** Upper gastrointestinal ultrasonography. (a) Doctor manually identifies early cancer lesions. (b) CNN model identifies early cancer lesions. (c) Cascade RCNN identifies early cancer lesions.

**Figure 6:** Comparison of lesion recognition accuracy between traditional CNN model group and Cascade RCNN model group (^∗^represents the statistical difference between the two groups, *P* < 0.05).

**Figure 7:** Comparison of lesion recognition recall rate between traditional CNN model group and Cascade RCNN model group (^∗^represents the statistical difference between the two groups, *P* < 0.05).

**Figure 8:** DSC comparison of lesion recognition between traditional CNN model group and Cascade RCNN model group (^∗^represents the statistical difference between the two groups, *P* < 0.05).

**Figure 9:** Comparison of lesion recognition learning rate between traditional CNN model group and Cascade RCNN model group (^∗^represented the statistical difference between the two groups, *P* < 0.05).

**Figure 10:** Comparison of lesion recognition number of iterations between traditional CNN model group and Cascade RCNN model group (^∗^represents the statistical difference between the two groups, *P* < 0.05).

**Figure 11:** Comparison of lesion recognition predicting speed between traditional CNN model group and Cascade RCNN model group (^∗^represents the statistical difference between the two groups, *P* < 0.05).

**Figure 12:** Ultrasonic image characteristics and endoscopy in patients with early upper gastrointestinal cancer. (a) Endoscopy in patients with early upper gastrointestinal cancer. (b) Ultrasonic image characteristics of patients with early upper gastrointestinal cancer.

**Figure 13:** Number of positive and negative endoscopic predictions, positive and negative pathological tissue detection in traditional CNN model group (^∗^represented the statistical difference among groups, *P* < 0.05).

**Figure 14:** Number of positive and negative endoscopic predictions, positive and negative pathological tissue detection in Cascade RCNN model group (^∗^represents the statistical difference among groups, *P* < 0.05).

**Figure 15:** Number of positive and negative endoscopic predictions, positive and negative pathological tissue detection in control group (^∗^represents the statistical difference among groups, *P* < 0.05).

**Figure 16:** Comparison of true positive rate of lesions in three groups (^∗^represented the statistical difference among groups, *P* < 0.05).

**Figure 17:** Comparison of true negative rate of lesions in three groups (^∗^represented the statistical difference among groups, *P* < 0.05).

**Figure 18:** Comparison of positive predictive value of lesions in three groups (^∗^represented the statistical difference among groups, *P* < 0.05).

**Figure 19:** Comparison of negative predictive value of lesions in three groups (^∗^represented the statistical difference among groups, *P* < 0.05).

## Data Availability

The data used to support the findings of this study are available from the corresponding author upon request.
